# Effect of Remote Control Augmented Reality Multimedia Technology for Postoperative Rehabilitation of Knee Joint Injury

**DOI:** 10.1155/2022/9320063

**Published:** 2022-05-27

**Authors:** Lingfeng Li

**Affiliations:** Department of Orthopaedics, Shanghai Fifth People's Hospital, Fudan University, Shanghai 200240, China

## Abstract

This study was aimed at exploring the application value of augmented reality (AR) in postoperative rehabilitation training for patients with knee joint injury. 40 patients who underwent knee joint injury surgery were selected as the research objects, and the patients were randomly divided into two groups: an experimental group (20 cases) and a control group (20 cases). Patients in the experimental group were treated with AR-based rehabilitation methods, while those in the control group were treated with traditional rehabilitation methods. Afterwards, the two groups of patients were compared with various indicators such as pain value, swelling, structural and functional recovery, time to complete weight bearing, time to return to work, and X-ray examination results. The main evaluation tools used were Hospital for Special Surgery (HSS) score and Visual Analogue Scale (VAS) score. The results showed that after six weeks, the HSS score of the control group was 82.88 ± 3.07, and the HSS score of the experimental group was 85.46 ± 3.21. The difference between the two groups was statistically significant (*P* < 0.05). After three months, the HSS score of the control group was 89.96 ± 3.76, and that of the experimental group was 93.21 ± 4.33. The difference between the two groups was statistically significant (*P* < 0.05). There was a significant difference in pain scores between the two groups at 7 days (3.81 ± 0.48 vs. 5.06 ± 0.66) and 14 days (2.03 ± 0.45 vs. 3.61 ± 0.63) after surgery, with statistical significances (*P* < 0.05). There were statistically significant differences between the two groups in terms of time to complete weight bearing (7 ± 0.87 weeks vs. 8.82 ± 0.88 weeks) and time to return to work (8.69 ± 0.94 vs. 9.93 ± 0.88 weeks) (*P* < 0.05). One month after surgery, the X-ray examination results of both groups showed recovery. The AR-based rehabilitation training system showed a good application effect and prospect in the postoperative structural and functional recovery of patients with knee joint injury.

## 1. Introduction

The knee joint is one of the largest and most complex joints in the human body. After a knee joint injury, the injury end can directly affect the functional activities of the knee joint, which is mainly manifested as limited knee joint movement and disuse atrophy of the muscles around the knee joint or arthrogenous muscle inhibition (AMI) [1]. The injury itself can make serous fibrous exudate and fibrin in the interstitial space deposited in the knee joint cavity, resulting in fibrous adhesions [2]. Long-term immobilization can cause disuse muscle atrophy, osteoporosis, etc. and can also cause articular cartilage nutritional disorders, atrophy, and fibrosis. Immobilization also causes synovial sacs to dry up and adhere, resulting in joint cavity stenosis [3]. It has been clinically confirmed that the joint immobilization time of 1 month and 3 months is negatively correlated with the recovery of knee flexion function. Many patients cannot receive early rehabilitation after joint surgery and trauma, so the incidence of knee joint dysfunction is high [4]. The main reason for knee joint adhesion is postoperative lower extremity immobilization, and knee joint dysfunction caused by knee joint adhesion can seriously affect the patient's ability to perform activities of daily living [5].

In recent years, with the development and progress of the concept of rehabilitation, the importance of early functional training after injury surgery has been gradually recognized and accepted [6]. However, with the rehabilitation training system based on virtual reality technology, patients need to face a different reality and virtual world every day, which is prone to anxiety. Therefore, none of these methods can achieve the expected rehabilitation effect. In this context, augmented reality (AR) was introduced into the field of rehabilitation. AR system shows many advantages such as three-dimensional registration, virtual and real combination, and real-time interaction, so it has been widely used in industries, military, cultural relic protection, games, and other fields [7]. Combining the AR technology with the principles of rehabilitation medical treatment can create a complex scene of the virtual reality and reality of the patient based on the physiological structure and movement of the knee joint, which is very beneficial to promote the recovery of damaged joints. And in rehabilitation therapy, repeated training of movements based on the patient's daily life can mobilize neurons with residual functions to participate in activities, which can promote the brain's nerve center to repeatedly correct and modify the quality of movements [8]. This is very beneficial to the structural and functional restoration of injured joints. In addition, rehabilitation training and rehabilitation assessment can play a mutually reinforcing relationship. Based on the patient's training data, it excavates the training behavior behind it and intelligently evaluates the patient's training effect and rehabilitation situation while providing reference and basis for the formulation of the next stage of training plan. In summary, AR technology has shown a strong application prospect in postoperative rehabilitation of bones and joints. At present, scholars have applied augmented reality technology to the rehabilitation training of joint injuries. For example, some scholars have developed an AR-based rehabilitation evaluation and training system for wrist joint ulna-radial deviation and carried out verification experiments. The results of the study showed that this method can effectively help patients with wrist joint ulnar deviation radial deviation rehabilitation training [9]. However, there are few relevant studies on the application of AR ankle rehabilitation training.

In this study, 88 patients who underwent knee joint injury surgery were selected as the research objects. The patients were randomly divided into two groups: an experimental group and a control group. Patients in the experimental group were treated with AR-based rehabilitation after the surgery, and those in the control group were treated with traditional rehabilitation. The efficacy of the two groups was observed and compared before training (i.e., 15 days after surgery) and four weeks after training. This study was expected to provide reference and basis for the treatment of clinically related diseases.

## 2. Materials and Methods

### 2.1. Research Objects

In this study, 40 patients who underwent knee joint injury surgery in the hospital from March 2019 to October 2020 were selected as the research objects. All patients were divided into three types A, B, and C according to the Danis-Weber classification. The detailed classification method is shown in Table 1. The experimental group included 8 male patients and 12 female patients, with an average age of 33.6 ± 8.11 years old, an average weight of 68.7 ± 8.33 kg, and an average hospital stay of 13.88 ± 1.31 days. The control group included 10 male patients and 10 female patients, with an average age of 31.8 ± 7.36 years old, an average weight of 67.41 ± 6.37 kg, and an average hospital stay of 14.62 ± 1.23 days. There was no significant difference in general data between the two groups of patients, and they were comparable. The patients were randomly divided into two groups: experimental group (20 cases) and control group (20 cases). Patients in the experimental group were treated with AR-based rehabilitation after the surgery, and those in the control group were treated with traditional rehabilitation. The informed consents were obtained from patients and met this study had been approved by the ethics committee of hospital.

The diagnostic criteria of knee joint injury were set as follows: patients with clear history of knee joint trauma; patients with knee joint injury, injuries with obvious movement, and injuries such as deformity and bone fricative. X-ray film showed that the knee joint space changed. CT clearly showed the injury displacement from all angles. Inclusion criteria were determined as follows: patients who met the above-mentioned diagnostic criteria for knee joint injury; patients with injury time within one week; patients with no surgical contraindications; and patients with complete information. Patients who met below criteria had to be excluded: those who did not meet the inclusion and diagnostic criteria; patients with pathological injuries and open injuries; patients with tibial pilon injuries; patients with soft tissue necrosis before and after surgery; and patients suffering from serious primary diseases of the heart, brain, stem endocrine, and hematopoietic system or mental illnesses so that they could not cooperate the experiment.

### 2.2. AR-Based Rehabilitation Training Technology

AR-based rehabilitation training technology mainly includes three parts: real scene training data acquisition, virtual scene construction, and virtual and real fusion. The detailed process was as follows:

Real scene training data acquisition was the prerequisite for the fusion of virtual and real. Firstly, it should determine the activity plane. The ulnar movement angle of the knee joint rotating around the *z* axis can be abstracted into a model,

AR-based rehabilitation training technology mainly includes three parts: real scene training data collection, virtual scene construction, and virtual reality fusion. The specific process was as follows. The collection of real scene training data was the premise of virtual-real fusion. First, it should determine the active plane. The ulnar motion angle of the knee joint rotating around the *z* axis can be abstracted into a model, as shown in Figure 1. The dotted line indicated the initial position, and the solid line marked the rotated position.

The left knee joint was taken as an example. It was assumed that at the moment *t*, the movement plane of the left knee joint was *δ*(t); then, the movement angle of the left knee joint a(t) computing method is shown in below equation:

(1) $$\begin{array}{c} \text{a}\left(\text{t}\right)=\text{data}\_\text{z}\left(\text{t}\right)-\text{data}\_\text{z}\left(0\right). \end{array}$$

Below equation could be obtained when it was rotated forward:

(2) $$\begin{array}{c} \text{data}\_\text{z}\left(\text{t}\right)>\text{data}\_\text{z}\left(0\right). \end{array}$$

Then, equation (3) below could be obtained:

(3) $$\begin{array}{c} \text{a}\left(\text{t}\right)>0. \end{array}$$

Below equation could be obtained when it was rotated in reverse:

(4) $$\begin{array}{c} \text{data}\_\text{z}\left(\text{t}\right)<\text{data}\_\text{z}\left(0\right). \end{array}$$

At this time, below equation could be satisfied.

(5) $$\begin{array}{c} \text{a}\left(\text{t}\right)<0. \end{array}$$

Afterwards, the knee joint motion angle model can be abstracted according to the rotation direction and angle of the rotator.

The virtual scene construction was given as follows. Based on AR exercise therapy scene modeling analysis (taking the left knee joint as an example), the plane model of the left knee joint exercise therapy is shown in Figure 1.

The phase goal *θ*(t) was given as follows from the moment *t*:

(6) $$\begin{array}{c} \theta \left(\text{t}\right)=\text{data}\_\text{zz}\left(\text{t}\right)\left(\theta \left(\text{t}\right)<60^{{}^{\circ}}\right). \end{array}$$

The best result ROM in the latest rehabilitation training was given as follows:

(7) $$\begin{array}{c} \text{a}\left(\text{t}\right)=\max\left\{\beta \left(\text{t}-1\right)\right\}. \end{array}$$

When *β*(t) − *α*(t) > 0, it meant that the knee joint had improved after rehabilitation training, on the contrary (*β*(t) − *α*(t) < 0), it meant that it had declined; *θ*(t) − *β*(t) > 0 meant that the patient had not completed the phase goal and required training, on the contrary (*θ*(t) − *β*(t) < 0), it meant that the patient had completed the phase task, and it also needed to be combined with other indicators for comprehensive rehabilitation training assessment. *β*(t) represented the angle of completion of the patient.

The steps of virtual and real fusion can be briefly summarized as follows. Firstly, the acquisition of relevant information for this training, such as the acquisition of training joints and duration and target angle. Secondly, the relevant parameters of the virtual scene were calculated and the initial modeling of the virtual scene was performed based on the rehabilitation training data information. Thirdly, the sensor was adopted to obtain the angle value of the knee joint in the real environment, and the angle value of the activity plane and joint movement angle value were saved. Fourthly, corresponding rotation direction and angle of the virtual object from the intermediate value obtained in step (3) were calculated, and the relevant parameters of virtual scene modeling were updated. Fifthly, the virtual objects were modeled based on real wrist motion images, and then, the fusion scene of virtual and reality was shown to the patient to guide their training.

### 2.3. Rehabilitation Training Method for Two Groups of Patients

Rehabilitation training method for patients in the experimental group was described as follows. In the early stage of training, the knee joint was in a sticky state and the nearby muscles and soft tissues were also paralyzed. At this time, if the training method was not appropriate, it was very easy to cause secondary joint damage. Therefore, in the initial stage of rehabilitation training, only exercise therapy was performed, and a virtual knee joint was constructed in the exercise therapy to drive the real knee joint to carry out small-angle training. At the same time, the real training data and information would be transmitted into the virtual scene and trigger the rerendering of the virtual scene and then guide the patient to carry out a larger angle and deeper training. In the middle and late stages of rehabilitation, it was necessary to add occupational therapy on the basis of exercise therapy training and render aircraft roaming scene games in occupational therapy, realizing the training of knee joint compound movement. The difficulty of the scene can be changed by adjusting the initial altitude of the aircraft. The system also sets the limit angle of the moving platform to protect the patient from exceeding the maximum angle during training.

The training method of the control group was described as follows. After the surgery, the affected limb was raised above the level of the heart, and the dressing was changed and sutures were removed routinely. On the first postoperative day, the patients were instructed to perform passive ankle motion exercises. On the third day after operation, active ankle exercise was performed, with dorsiflexion and plantar flexion 3-5 times each. In the first week after operation, the patient was asked to move on the ground with crutches, but the affected limb did not touch the ground. According to the local condition after the surgery, the patient's activity intensity and activity volume should be appropriately increased based on the imaging situation. In the second week after the surgery, the patient was required to continue to perform functional activities on the bed without weight-bearing exercises if the affected area was still swollen or tender. If the affected area was not swollen and the tenderness was not obvious, the patient was asked to walk on the toes with crutches on the ground. In the fourth week after the surgery, it should continue to practice the ankle joint function, exercise 3 times a day, 6-8 times each time; follow the X-ray situation; or continue to practice with or without weight bearing. After the sixth week after surgery, routine X-ray examination was performed, and functional exercise methods were adjusted in time according to the patient's symptoms, signs, and X-ray performance. If there was callus growth at the fracture end, the affected limb was allowed to perform weight-bearing exercise with crutches.

### 2.4. Observation Indicators

The commonly used clinical HSS knee score was selected to analyze the patients' knee joint at 6 weeks and 3 months after surgery (Table 2).

The Visual Analogue Scale (VAS) (Figure 2) was adopted to assess the degree of postoperative knee joint pain. 0 meant no pain; 10 cm meant the most painful; 1~3 cm meant mild pain; 4~6 cm meant moderate pain; and 7~10 cm meant severe pain.

The patient was informed the follow-up requirements in detail and rechecks X-ray examinations every week after 4 weeks after the operation. According to the patient's local condition and imaging conditions, it could guide the patient to perform functional exercises and recheck on time until the patient fully tolerates the weight bearing. If there was no obvious displacement of the injury end on the X-ray film and there was formation of callus, the patient was allowed to bear weight. In addition, the time to complete weight bearing and time to return to work time of patients were observed and recorded.

### 2.5. Statistical Methods

SPSS 22.0 statistical software was used for data analysis. Measurement data were expressed as mean ± standard deviation ($\overset{-}{x}\pm s$). Comparison between groups was performed by *t*-test; comparison within groups was performed by analysis of variance; and count data was used by *χ*^2^ test. *P* < 0.05 meant the difference was statistically significant.

## 3. Results

### 3.1. The General Information of Patients

The general information of the patient is shown in Table 3. Analysis of Table 3 showed that the experimental group included 8 male patients and 12 female patients; the average age was 33.6 ± 8.11 years old, the average weight was 68.7 ± 8.33 kg, the average hospital stay was 13.88 ± 1.31 days, and the circumference of the uninfected knee joint was 23.93 ± 0.69 cm. Patients in the control group included 10 male patients and 10 female patients, the average age was 31.8 ± 7.36 years old, the average weight was 67.41 ± 6.37 kg, the average length of hospital stay was 14.62 ± 1.23 days, and the circumference of the uninfected knee joint was 25.63 ± 0.76 cm. There was no statistically significant difference between the two groups of data. Therefore, there was comparability between the two groups of patients.

### 3.2. Comparison on Postoperative Relief between the Two Groups

As shown in Figure 3, 14 days after the surgery, 5 cases were markedly effective, 15 cases were effective, and 0 cases were ineffective in the experimental group; while 6 cases were markedly effective, 11 cases were effective, and 3 cases were ineffective in the control group. There was a significant difference between the effective number and the ineffective number between the two groups (*P* < 0.05).

### 3.3. Comparison of Knee HSS Scores between the Two Groups

Knee HSS scores were performed at 6 weeks and 3 months after surgery. The results showed that after 6 weeks, the HSS score of the control group was 82.88 ± 3.07, and the HSS score of the experimental group was 85.46 ± 3.21, the difference between the two groups was statistically significant (*P* < 0.05). After three months, the HSS score of the control group was 89.96 ± 3.76, and that of the experimental group was 93.21 ± 4.33, the difference was statistically significant (*P* < 0.05). The overall score of the experimental group was higher than that of the control group, and the postoperative recovery was better. The total HSS scores of the two groups are shown in Figure 4.

### 3.4. Comparison on Postoperative Pain Values between the Two Groups

Figure 5 shows the comparison of the pain values between the two groups of patients at various time periods after surgery. Analysis of Figure 6 showed that there was no significant difference in the pain value between the two groups of patients on the three days after the surgery. The patients on the 7th day after the surgery (3.81 ± 0.48 vs. 5.06 ± 0.66) and the 14th day after the surgery (2.03 ± 0.45 vs. 3.61 ± 0.63) were significantly different (*P* < 0.05).

### 3.5. Comparison on Time to Complete Weight Bearing and Time to Return to Work of Patients in Two Groups

The comparison results of time to complete weight bearing and time to return to work between the two groups of patients are shown in Figure 6. Analysis of Figure 7 showed that the time to complete weight bearing of the experimental group was 7 ± 0.87 weeks, and the time to complete weight bearing of the control group was 8.82 ± 0.88 weeks. The time to return to work in the experimental group was 8.69 ± 0.94 weeks, and the time to return to work in the control group was 9.93 ± 0.88 weeks. The differences between the two groups of time to complete weight bearing and time to return to work were statistically significant (*P* < 0.05).

### 3.6. Imaging Data of Typical Cases

Figure 7 shows the X-ray examination results of the knee joint of the two groups of patients. With the continuous deepening of the training level, the knee joint structure of the two groups of patients had recovered. In the same time period, the recovery of the knee joint of the experimental group was better than that of the control group.

## 4. Discussion

The knee joint is the largest trochlear joint in the human body with the most complex structural composition and function. The knee joint lacks soft tissue protection, and external forces can be directly transmitted to the bony tissue to cause knee joint injury [10]. Due to external fixation of the knee joint after the operation, the synovial fluid in the joint failed to circulate effectively, and the fibrin formed adhesions in the folds of the joint capsule, the synovial reflex, and the muscles. After 5 to 7 days of joint immobilization, the muscle abdomen will shorten, and after 3 weeks, the loose connective tissue around the joint will become dense connective tissue, the motor neuron recruitment will decrease, and the joint will be rigid [11]. In addition, braking causes articular cartilage dystrophy, atrophy, necrosis, fibrosis, synovial sac drying, disappearance of adhesions, and joint stenosis causing adhesions [12]. Surgical internal fixation creates conditions for injury healing and is the basis of comprehensive treatment. Immobilization is one of the main treatment measures after injury surgery. However, immobilization can cause pathological changes in the body's joint capsule, ligaments, muscles, and other tissues in terms of morphological structure, biochemistry, and biochemical mechanics and ultimately affect the function of joints and limbs [13]. In order to avoid knee joint dysfunction, a comprehensive treatment based on early functional activities has to be adopted [14].

In recent years, the Internet and computer technology have made rapid progress and development, and many new technologies have emerged. AR is currently a technology with relatively high attention. AR technology is a new technology developed on the basis of virtual networks, which can superimpose computer-generated virtual objects onto real scenes through display technology, so that the real environment and the virtual environment are integrated, and the effect of AR is further achieved. Virtual reality technology can construct a virtual environment similar to the real scene and can bring users real-time feedback during rehabilitation training [15]. To a certain extent, it enhances the fun of training and the enthusiasm of patients in training, but the virtual environment constructed by it is completely separated from the real scene. Therefore, if AR technology can be applied to rehabilitation training, it will be a breakthrough in the field of rehabilitation. At present, there are many research contents in related fields and certain achievements have been made. For example, some scholars have developed an AR-based rehabilitation evaluation and training system for wrist joint ulna-radial deviation and carried out verification experiments. The results of the study showed that this method can effectively help patients with wrist joint ulnar deviation radial deviation rehabilitation training [16]. But there are still some problems. For example, the equipment used in some studies is expensive and cannot be widely promoted in clinical practice, and the equipment used in some studies is too cumbersome and cumbersome to pass on, and the training scene is not immersive [17]. In addition, there is almost no relevant research on the application of AR ankle rehabilitation training. In response to the above problems, a knee joint resistance training system based on AR technology was proposed and applied to postoperative rehabilitation of knee joint injury patients. In addition, its training effect was compared with traditional rehabilitation methods. The results showed that, compared with traditional methods, the rehabilitation training method based on AR showed strong advantages in relieving postoperative pain and helping structural and functional recovery. In addition, the training method proposed in this study was more interesting, and the training enthusiasm of patients was significantly increased. At the same time, the cost was relatively low, and it can be said that it had a broad clinical application prospect.

## 5. Conclusion

In this study, a knee joint rehabilitation training system based on AR technology was proposed and a verification experiment was carried out. The results showed that, compared with traditional methods, the rehabilitation training method based on AR showed strong advantages in alleviating postoperative pain and helping structural and functional recovery. In summary, AR technology had a good clinical application prospect in rehabilitation training for patients with knee joint injury. Due to limited samples and space, this study was not comprehensive and in-depth enough. For example, when the effects of rehabilitation were evaluated, it only analyzed the pain relief, swelling, and structural and functional recovery. There were no statistics on the enthusiasm of the patients who were interested in training. In the future study and work, it will expand the sample to further comprehensively and in-depth study this issue.

## Figures and Tables

**Figure 1:** Knee joint exercise therapy rehabilitation training model.

**Figure 2:** VAS.

**Figure 3:** Comparison on postoperative relief between the two groups. ^∗^Compared with the control group, *P* < 0.05.

**Figure 4:** Comparison of KNEE HSS score between the two groups. ^∗^Compared with the control group, *P* < 0.05.

**Figure 5:** Comparison on postoperative pain value between the two groups. ^∗^Compared with the control group, *P* < 0.05.

**Figure 6:** Comparison on time to complete weight bearing and time to return to work of patients in two groups. ^∗^Compared with the control group, *P* < 0.05.

**Figure 7:** X-ray examination results of typical cases in two groups at each time period. Patient information of the experimental group: male patients aged 44.3 ± 9.3 years old, injury type A. Patient information of the control group: male patients aged 55.1 ± 11.4 years old, injury type B.

**Table 1:** The Danis-Weber classification results.

Type	Manifestation
A	
A1	Simple fibula fracture
A2	Combined medial malleolus fracture
A3	Combined medial and posterior fractures
B	
B1	Simple fibula fracture
B2	Combined medial injury
B3	Combined medial injury and posterolateral tibia fracture
C	
C1	Simple fibular shaft fracture
C2	Compound fibular shaft fracture
C3	Proximal fibula fracture

**Table 2:** HSS score of knee joint.

Item	Score
Pain	
No pain at anytime	30
No pain while walking	15
No pain while resting	15
Slight pain while walking	10
Slight pain while resting	10
Moderate pain while walking	5
Moderate pain while resting	5
Severe pain while walking	0
Severe pain while resting	0
Function	
Walking and standing unrestricted	12
Walk 1,000-2,000 m	10
Walk 200-1000 meters and stand for up to half an hour	8
Can go up stairs	5
Public transport	5
Walk less than 200 meters	4
Public transportation, support required	2
Can climb stairs, need support	2
Cannot walk	0
Activity level (maximum 18 points)	
Level 8	1
Muscle strength	
Excellent: fully able to resist resistance	10
Good: partly against resistance	8
Moderate: can drive joint movement	4
Bad: cannot drive joint movement	0
Flexion deformity	
No deformity	10
Less than 5 degrees	8
5~1 degrees	5
More than 10 degrees	0
Stability	
Normal	10
Slightly unstable, 0~5 degrees	8
Moderately unstable, 5~15 degrees	5
Severely unstable, more than15 degrees	0
Markdown items	
Single stick	-1
5 degrees of unbending stagnation	-2
Valgus every 5 degrees	-1×
Single crutches	-2
10 degrees of unbending stagnation	-3
Pronation every 5 degrees	-1×
Double crutch	-3
15 degrees of unbending stagnation	-5

**Table 3:** Comparison of general information of the two groups of patients (*n*, $\bar{x}\pm s$).

Item	Groups	
	Experimental group	Control group
Age (years old)	33.6 ± 8.11	31.8 ± 7.36
Weight (kg)	68.7 ± 8.33	67.41 ± 6.37
Circumference of the uninfected knee joint (cm)	23.93 ± 0.69	25.63 ± 0.76
Hospital stay (days)	13.88 ± 1.31	14.62 ± 1.23
Gender		
Males	8	10
Females	12	10
Injury site		
Left	13	12
Right	7	8
Type of injury		
B	11	8
C	9	12

## Data Availability

The data used to support the findings of this study are available from the corresponding author upon request.
